# Prediction of College Students' Sports Performance Based on Improved BP Neural Network

This article has been retracted.

**DOI:** 10.1155/2022/5872384

**Published:** 2022-08-08

**Authors:** Hengyao Tang, Guosong Jiang, Qingdong Wang

**Affiliations:** Computer School of Huanggang Normal University, Huanggang, Hubei 43800, China

## Abstract

Sports performance prediction has gradually become a research hotspot in various colleges and universities, and colleges and universities pay more and more attention to the development of college students' comprehensive quality. Aiming at the problems of low accuracy and slow convergence of the existing college students' sports performance prediction models, a method of college students' sports performance prediction based on improved BP neural network is proposed. First, preprocess the student's sports performance data, then use the BP neural network to train the data samples, optimize the selection of weights and thresholds in the neural network through the DE algorithm, and establish an optimal college student's sports performance prediction model, and then based on cloud computing, the platform implements and runs the sports performance prediction model, which speeds up the prediction of sports performance. The results show that the model can improve the accuracy of college students' sports performance prediction, provide more reliable prediction results, and provide valuable information for sports training.

## 1. Introduction

Nowadays, with the improvement of external material living standards and the popularization of network information, the overall physical quality of college students shows an obvious downward trend [1, 2]. The physical quality of the students is mainly assessed by the standard physical education results of the students in the physical education class in colleges and universities. Therefore, the high performance prediction of physical education results has become a key factor in the development of physical education curriculum and training by the Ministry of Education, and at the same time, in this context, a reasonable sports performance prediction method has gradually become a hot research issue in various universities [3, 4].

In essence, the prediction of students' PE scores can be regarded as a regression problem. Researchers have put forward many different methods for this problem, and the prediction has been completed based on students' physical fitness and simple statistical methods at first and gradually developed towards improved efficiency and accuracy [5]. Among many methods, the application of multiple linear regression model is not the best because of the interference of nonlinear factors in sports performance prediction. However, the method in view of BP proposed in literature [6] overcomes the interference of nonlinear factors in the prediction and optimizes the prediction performance, but the convergence speed is slow, and the result is easy to be a local optimal solution. If the parameters that have great influence on the result, such as threshold value and weight value, are set improperly, the prediction of the result will also be affected. In order to solve the parameter problem of neural network effectively, some scholars applied genetic algorithm and particle swarm optimization algorithm to determine the key parameters of neural network and realized the purpose of improving the accuracy of grade prediction. Because genetic algorithm and particle swarm optimization algorithm easily fall into local optimal solution and usually can only get suboptimal solution, it is difficult to calculate the global optimal solution of the main parameters such as threshold value and weight value, which makes the learning time of neural network long and the structure complex, thus affecting the modeling effect of sports performance prediction. The prediction method based on particle swarm optimization support vector machine proposed in literature [7] optimized the prediction accuracy and achieved good prediction effect. Although the sports performance prediction method based on firefly optimized neural network proposed in literature [8] improves the prediction accuracy, it is difficult to be adopted and applied in universities due to the high complexity of the established model.

With the continuous development of information processing technology, the processing and analysis of big data information through cloud computing platform have become the current technology development trend. Cloud computing platform can effectively improve data parallel processing capability and computing speed, enhance data processing efficiency, and optimize based on differential evolution algorithm. The neural network model can better model and analyze the prediction of sports performance. The results show that the model in this paper can improve the prediction accuracy of sports performance, and the prediction results are more reliable [9, 10].

## 2. BP and DE

### 2.1. BP

Backpropagation (BP) neural network is a highly complex and nonlinear dynamic analysis system proposed by Rumelhart and McClelland in 1986. It forms an interconnected network structure through various independent units [11–15]. The neural function learns the data samples, establishes the connection weights and thresholds between the units, and then deals with complex nonlinear problems without specific functional forms [16–18]. It is a multilayer feedforward neural network with forward signal propagation and error backpropagation. The training process of BP neural network can be divided into two parts: forward propagation and backpropagation. It forward-propagates from the input layer through the hidden layer to the output layer and then backpropagates from the output layer to the hidden layer and then to the input layer. In the training process, the forward propagation is from the input layer through the hidden layer, and then to the output layer. Backpropagation is from the output layer to the hidden layer, and then to the input layer [19–21]. In the process of neural network training, the trained model is forwarded to obtain the predicted value, and the weight is corrected according to the error between the actual value and the predicted value. If the error exceeds the set threshold, the error is backpropagated [22–27]. After the neural network is initialized, the parameters of the entire network are adjusted through backpropagation, and the weights and thresholds of neurons are continuously corrected and learned until the output error reaches the expected result, and the neural network training is considered complete.

One or more neuron layers are set up BP to compute data; each neuron layer can have multiple nodes. Double hidden layer has the advantage of fast classification speed, so this paper adopts double hidden layer network structure. By adjusting the weight matrix and error feedback between each layer, the desired effect is achieved. The BP with double hidden layer has improved data parallel processing and accuracy, as shown in Figure 1.

The input vector of BP is *K*=(*k*_1_, *k*_2_, *k*_3_, ⋯,*k*_*n*_)^*T*^, and the weight matrix of input layer and hidden layer is *S*_*ni*_ (1 < *n* < *N*, 1 < *i* < *I*), the weight matrix is *W*_*ij*_ (1 < *i* < *I*, 1 < *j* < *J*), the output vector of the first hidden layer is *B*=(*b*_1_, *b*_2_, *b*_3_, ⋯,*b*_*n*_)^*T*^, the threshold value on node *i* of the second hidden layer is *θ*_*i*_, the threshold value on node *j* of the second hidden layer is *C*=(*c*_1_, *c*_2_, *c*_3_, ⋯,*c*_*n*_)^*T*^, the weight matrix is *W*_*jn*_, the output vector of the output layer is *D*=(*d*_1_, *d*_2_, *d*_3_, ⋯,*d*_*n*_)^*T*^, the threshold value on node *N* of the output layer is *θ*_*n*_, and *f*(*x*) is the activation function. Input *n*-dimensional vector *A*, and then the output of node *i* of the first hidden layer is

(1) $$\begin{array}{c} b_{i}=f\left(\sum_{i=1}^{m}w_{mi}a_{m}-\theta_{i}\right). \end{array}$$

The output of node *J* of the second hidden layer is

(2) $$\begin{array}{c} c_{j}=f\left(\sum_{j=1}^{I}w_{ij}b_{i}-\theta_{j}\right). \end{array}$$

The output result of the *N*TH node in the output layer is

(3) $$\begin{array}{c} d_{n}=f\left(\sum_{n=1}^{J}w_{jm}c_{j}-\theta_{n}\right). \end{array}$$

In order to improve the convergence speed of BP neural network, the input data is normalized to reduce the range of change and improve the flexibility of interval selection. The formula is as follows:

(4) $$\begin{array}{c} t_{i}^{\prime }=\frac{t_{i}-t_{\min}}{t_{\max}-t_{\min}}, \end{array}$$

where *t_i_′* is the input value of the neural network, *t_i_* is the normalized value of the interval set [0, 1], tmin and tmaxare the minimum and maximum values of the sample, respectively.

The activation function is as follows:

(5) $$\begin{array}{c} f\left(x\right)=\frac{1}{1+e^{-x}}. \end{array}$$

### 2.2. DE

Differential evolution algorithm (DE) is a random search heuristic technology based on group differences. It is a new and efficient technology. DE algorithm is developed based on genetic algorithm. Similar to genetic algorithm, it has mutation, crossover, Select, and other operations, but the implementation is simple, and the convergence speed is fast. For the traditional BP neural network, there are generally problems such as local minima, slow convergence speed, and sometimes oscillation or even divergence in the entire calculation process. In order to overcome its limitations, the differential evolution algorithm (DE) is introduced into the traditional BP neural network to optimize the initial weights and thresholds of the network, which can make it have better nonlinear mapping ability and improve its prediction accuracy.

The overall structure of the differential evolution algorithm is similar to the genetic algorithm, by simulating the evolution of biological populations and iterating repeatedly, so as to retain the individuals that meet the adaptive conditions. The DE algorithm retains the global search ability of the genetic algorithm. It adopts the form of real number coding, the mutation method based on the difference principle, and the one-to-one competition survival mode, which greatly simplifies its calculation process. It has been successful in many fields.

The process of DE-DNN network model is as follows:

#### 2.2.1. DE Algorithm Initializes the Population

Determine the population size *m*, each individual is an *N*-dimensional vector, and the initial population can be expressed as the following formula:

(6) $$\begin{array}{c} X_{t}\left(0\right)=X_{t1}\left(0\right)+X_{t2}\left(0\right)+\cdots +X_{tj}\left(0\right), \end{array}$$

where the *t*-th individual of *X*_*t*_(0) generates 0, the JTH gene of the *t*-th individual of *X*_*tj*_(0) generates 0, *t* = 1, 2, ... , *M*.

#### 2.2.2. Variation of DE Algorithm

In the KTH iteration, for individual *X*_*t*_(*k*) = (*X*_*t*1_(*k* + *X*_*t*2_(*k*)+ ... + *X*_*tn*_(*k*)), a no. 1 intermediate vector *L*_*t*_(*k*) is generated as follows: three individuals *X*_*y*1_(*k*), *X*_*y*2_(*k*) and *X*_*y*3_(*k*) are randomly selected from the population, and *y*_1_ ≠ *y*_2_ ≠ *y*_3_, and then, the following equation can be obtained:

(7) $$\begin{array}{c} F_{t}\left(k\right)=X_{y1}\left(k\right)-E*\left(X_{y2}\left(k\right)-X_{y3}\left(k\right)\right), \end{array}$$

where ∆ = *X*_*y*2_(*k*) − *X*_*y*3_ (*k*) is the difference vector.

E is the scaling factor, which is used to control the influence of the difference vector and is generally between [0, 1].

In Figure 2, it can be intuitively seen that the variation vector *F*_*t*_(*k*) is constructed in the two-dimensional parameter space.

#### 2.2.3. DE Algorithm Crossover Operation

In the *K*TH iteration, each individual crosses with the first intermediate vector it generates. Specifically, for each of the same components, the first intermediate vector is selected with a certain probability, and the second intermediate vector *S*_*t*_(*k*) is generated. Each component of *S*_*t*_(*k*) is calculated according to the following formula:

(8) $$\begin{array}{c} S_{tj}\left(k\right)=\left\{\begin{array}{cc} F_{tj}\left(k\right), & rand\left(0,1\right)\leq P,\\ X_{tj}\left(k\right), & \text{else}, \end{array}\right) \end{array}$$

where *P* is the crossover probability, *F*_*tj*_(*k*) is a gene in the first intermediate vector, and *X*_*tj*_(*k*) is a gene in the original self.

#### 2.2.4. DE Algorithm Selection Operation

In this process, according to the value of fitness function, the second intermediate vector *S*_*t*_(*k*) and the original vector *X*_*t*_(*k*) with higher fitness of each individual are selected for the next generation in the *K*TH iteration, so as to make the population evolve to the optimal solution. The selection method is as follows:

(9) $$\begin{array}{c} X_{t}\left(k+1\right)=\left\{\begin{array}{cc} S_{t}\left(k\right), & f\left(S_{t}\left(k\right)>X_{t}\left(k\right)\right),\\ X_{t}\left(k\right), & \text{else}, \end{array}\right) \end{array}$$

After this step is completed, the differential evolution operation is continued until the number of iterations or fitness function is satisfied, and the algorithm stops.

### 2.3. Building a Cloud Computing Platform

Cloud computing platform is a new type of platform with multiuser shared infrastructure, which uses the Internet to send a large amount of storage and computing processing programs to distributed computers and provides application services for computers, enabling users to switch required resources to applications, Access the computing and storage systems in the cloud computing platform according to individual needs. The sports performance prediction model established above is packaged through MATLAB software and deployed to windows azure using the windows live developer portal. The cloud computing platform architecture is built through the above steps, as shown in Figure 3. The platform includes an infrastructure layer, a platform layer, and an application layer. The infrastructure layer is used to provide basic management applications of the cloud computing platform to users through the Internet. The infrastructure layer includes functions such as user security settings, permission settings, and connection between computers and servers. The platform layer is used to provide users with a server platform through the Internet, and the sports performance prediction model is placed in the platform layer. The cloud computing service provider data center predicts the user's required sports performance through the sports performance model and displays the results of different sports performance predictions in colleges and universities through the application layer to the user interface.

### 2.4. Operation Mode of Cloud Computing Platform

The cloud computing platform balances the load of each distributed computer through the task allocation and scheduling of the main target and effectively improves the processing efficiency. Abstractly integrate web services through various technologies in the cloud computing platform until an indivisible micro-linear unrelated service unit is obtained, send the service unit to multiple servers, and use the weakly related job scheduling algorithm, unrelated job scheduling algorithm, and strong asynchronous service request. The related job scheduling algorithm effectively improves the scheduling efficiency of asynchronous service requests.

The operation mode of cloud computing platform adopts sorting algorithm, and the operation mode is realized by bubble sort and insertion sort. When an abnormal task occurs in the sports performance prediction model, the above algorithm is used to deal with the abnormal task and allocate effective resources. The operation mode of the cloud computing platform is as follows:

1. The user opens the browser and uses the Internet to send out a sports performance prediction service request to the cloud computing platform, and the cloud computing platform uses the access agent to provide the user with sports performance prediction service information.
2. The user opens the browser and uses the Internet to send sports performance prediction service requests to each service provider in the cloud computing platform. When the cloud computing platform service provider receives too many sports performance prediction service requests, the cloud computing platform prompts an asynchronous service request. When the user who sends the sports performance prediction request is a VIP user, the cloud computing platform inserts the VIP user's sports performance prediction request before the queue through the insertion sorting method and preferentially processes the VIP user's sports performance prediction request, so that the VIP user can obtain the sports performance prediction service information. The time is earlier than that of other users; when the user who sends the sports performance prediction request is an ordinary user, after the VIP user's sports performance prediction request is processed, the ordinary user sends the request time sequence to process the sports performance prediction request and provide the sports performance prediction service information to general user.
3. When different users apply for the same sports performance prediction request, the application information is sent according to the above steps. When different or the same user applies for different sports performance prediction, the virtualization technology is used to make each server process the application information synchronously and decentralized.
4. Figure 4 shows the operation mode of the cloud computing platform when different users apply for the same sports performance prediction request. When different or the same user applies for different sports performance prediction requests, there are countless cloud computing platform operation modes that are the same as those in Figure 4. Run and process each request; that is, realize the common operation of most theoretical servers in the same physical server in the cloud computing platform.

### 2.5. Implementation Process of Cloud Computing Platform

The preparation of physical resources is the most important step in the implementation process of the cloud computing platform. In the cloud computing platform, the service provider data center uses the sports performance prediction model to predict the sports performance, which is the physical resource preparation process of the platform. The specific implementation process of the cloud computing platform is as follows:

In the cloud computing platform, the service provider data center uses the sports performance prediction model to predict sports performance and sends the predicted data to the application layer resource platform through virtualization technology. According to the performance prediction requirements of different sports performance items applied by users, different sports performance prediction results are allocated to realize different user prediction requirements. When the user needs are the same, the same sports performance prediction result is sent to the user to meet the user's prediction needs. The implementation process of sports performance prediction based on the cloud computing platform is shown in Figure 5.

#### 2.5.1. Processor Structure

The integration and processing of physical layer information are all implemented based on processors. In order to ensure the efficient and complete integration of construction engineering information, Advanced RISC Machine (ARM) processors are used in this paper. The functions of information acquisition, digital converter (AD), serial port, and external connection interface are built on ARM to realize the integrated processing of physical layer information. When the processor performs information integration processing, the interaction and communication of information are completed based on the VXI bus. After implementing the relevant information integration control for the collected various construction project budget information, the Digital Signal Processing (DSP) chip is used to filter the information, compression, and other processing; the processed information is used for scheduling between two buses, namely, the LOCAAL bus and the PCI bus, the scheduling between the two needs to be completed according to the interface circuit, and the clocks are constructed on the PCI and the local bus, respectively, to complete the interrupt reset.

#### 2.5.2. AD Submodule

During the execution of the processor, the collection and integration of the construction project budgetary information are completed through the AD submodule. In this paper, the STM32 chip is used as the information acquisition of the AD submodule of the processor, and the D/A converter is used to convert it into a digital signal and input it to the information processing terminal to realize the integrated processing and online processing of the construction engineering budget information mobilize.

#### 2.5.3. Local Database

The local database is used by the physical layer to realize the storage of integrated information. In this paper, the parallel structure is used to construct the database of this article to ensure the rationality of the distribution of information to the client and the server, and to ensure the efficient transmission of information. In order to improve the integration of the database, two technologies, TLXT1 and J2MAT, are integrated into the database construction process. At the same time, a logical collection of data is established in the database to realize data caching and analysis. The generation of logic is mainly based on the data allocation chip, which can reduce the amount of information cached during operation and achieve efficient storage. The database can complete the caching and analysis of information through the data allocation chip, which assigns the corresponding logical characters of the analyzed information to generate logical information codes. In the process of receiving information, the database needs to ensure the completeness of its receiving. The information receiving rate is

(10) $$\begin{array}{c} R=\frac{V_{i}}{I_{i}}\times P. \end{array}$$

In the formula, information bandwidth and outgoing coefficient are *V*_*i*_, *I*_*i*_, and all belong to the *i*-th frequency; *P* represents the maximum efficiency of communication.

## 3. DE-BP Neural Network Prediction Model

Differential evolution algorithm has a strong ability to optimize complex functions. For the initial weight and random threshold problems, DE algorithm is used to optimize and find the optimal weight and threshold. The algorithm process is as follows: firstly, the initial population of the algorithm based on the initial weight and threshold value is determined, and then the population is mutated, crossed, and selected. The fitness value is taken as the evaluation method of the current population to find the best individual in the population. When the output of the neural network is lower than the target error, the training process is terminated. The training process of DE-BP model is shown in Figure 6.

**Step 1 .**

Initialize all network parameters (related parameters of BP and DE);

**Step 2 .**

Initialize weights and thresholds;

**Step 3 .**

Initialize the fitness value, input the processed data into the model for training, and then take the calculated error mean value as the fitness value;

**Step 4 .**

Mutation, crossover, and selection are carried out to generate a new generation of individuals.

**Step 5 .**

Calculate the fitness value of new individuals;

**Step 6 .**

Check whether the completion conditions are met. If yes, go to the next step. If no, perform Step 4 again.

**Step 7 .**

Train the prediction model of college students' SPORTS results based on DE-BP.

## 4. Experimental Results

In order to verify the validity and superiority of the prediction of college students' sports performance based on DE-BP neural network proposed in this paper, the sports performance of students in a certain school is taken as the experimental object, the 100 m running results of 500 students are selected as the sample data, and the training set is 400 students. Student performance: train the model to obtain the optimal student sports performance prediction model, and then build a cloud computing platform, use the sports performance prediction model in the platform layer of the cloud computing platform to predict the sports performance, and use the different operation modes of the cloud computing platform to connect users. The required sports performance prediction results are sent to the user interface, and the test set is 100 people to test the predictive ability of the model.

In the DE algorithm, the parameter population size is initially set to 50, the scaling primer *E* is set to 0.5, and the maximum number of iterations is 100.

Figure 7 can conclude that the fitness value changes in model fitness value at the beginning of the iteration is bigger and has not found the population of the optimal solution algorithm, and it can be seen that, in the DE-BP optimization model in the iteration number of up to 20 times or so and the local search algorithm on a small scale, fitness values tend to be stable.

Through the trained model, 100 students are selected for testing, among which 20 students are selected. The predicted result of 100M and the real value as well as the error between them are shown in Figure 8.

The difference between the predicted value and the measured value is shown in Figure 7. By analyzing the predicted results of the 100-meter run, it can be seen that the predicted value is very close to the measured value, the difference between the two has high coincidence accuracy, and the error range is compared. It can be seen that, by using the DE optimization algorithm to adjust the weights and thresholds of the BP neural network, a better prediction model for college students' grades is established. The results show that the prediction results of the DE-BP model are reliable.

In order to analyze the superiority of DE-BP neural network in sports performance prediction results, multiple linear regression, GA-BP neural network, and PSO-BP neural network were selected for comparative experiments, and prediction accuracy, root mean square error, and percentage error were selected as performance comparisons. Parameters are used to evaluate the performance prediction results of the 100 m run, and the results are shown in Table 1. The performance comparison parameter solution formula is as follows:

(11) $$\begin{array}{c} RMSE=\sqrt{\frac{1}{n}\sum_{i=1}^{N}{\left(\hat{x}\left(i\right)-x\left(i\right)\right)}^{2}},\\ \text{MAPE}=\frac{1}{n}\overset{n}{\underset{i=1}{\sum }}\left|\frac{\hat{x}\left(i\right)-x\left(i\right)}{x\left(i\right)}\right|\times 100\%. \end{array}$$

In the formula, RMSE means root mean square error; MAPE means percentage error; *n* means the number of test samples.

We can get from the above table that, with the multiple linear regression model, the result has the lowest accuracy, indicating that the multiple linear regression is not suitable for the prediction of the 100-meter result, and the prediction error result is large, and the practical value is low. The prediction accuracy of GA-BP model and PSO-BP model is obviously better than that of multiple linear regression, indicating that BP network is a method with strong nonlinear modeling ability and can obtain better prediction results, but some students' prediction results are not ideal. The best prediction result is with DE-BP model, indicating that DE algorithm solves the problem that GA and PSO algorithms found difficult to obtain more ideal performance prediction results. The multiple linear regression model predicts that the RMSE value and MAPE value of the university's 100 m score are the highest. This is because the multiple linear regression model is more accurate in predicting the regular change trend, while the college 100 m running score is a nonlinear change trend. The regression model is difficult to solve accurately, so the prediction results have a large deviation. The RMSE value and MAPE value of the neural network model predicting the university's 100 m running performance are smaller than those of the multiple linear regression model, but significantly larger than those of the model in this paper. This is because the neural network model uses the empirical risk minimization algorithm for prediction, and it is more likely to occur in the prediction process. Fitting and other phenomena result in a large deviation between the predicted 100 m running performance and the actual performance. Using this model for prediction, the RMSE value and MAPE value of the university's 100 m grades were significantly smaller than those of the autoregressive sum model and the neural network model. This is because the model in this paper optimizes the BP neural network through the DE algorithm to establish a sports performance prediction model to achieve sports performance prediction. The model of this paper can better fit the characteristics of sports performance changes and effectively improve the prediction accuracy of 100 m running results.

Finally, additional experiments are conducted to verify the versatility of the model in this paper. The predictions for 1000 m run, marathon, triple jump, and shot put are performed, respectively. The predicted results are shown in Figure 9.

As shown in the figure, compared with the other three models, the model in this paper has higher prediction accuracy, and the prediction accuracy of other items is greater than 85%, which proves the strong versatility of the model in this paper.

## 5. Conclusion

College students' sports performance is an important reference data for analyzing college students' physical and sports conditions, and the prediction of college students' sports performance is the key basis for effective guidance for future teaching plans. The neural network has the disadvantages of slow convergence speed and missing the global optimal value. The differential evolution algorithm is used to optimize the neural network, and a prediction method of students' sports performance based on DE-optimized BP neural network is proposed. Firstly, preprocess the students' sports performance data, then use the BP neural network to train the data samples, and optimize the selection of weights and thresholds in the neural network through the DE algorithm to establish the optimal prediction model of college students' sports performance, which further improves the prediction performance and precision. The results show that the model can improve the accuracy of college students' sports performance prediction, provide more reliable prediction results, and provide valuable information for sports training.

## Figures and Tables

**Figure 1:** Structure diagram of BP.

**Figure 2:** Schematic diagram of variation vector construction.

**Figure 3:** Cloud computing platform architecture.

**Figure 4:** Cloud computing platform operating mode.

**Figure 5:** Implementation process.

**Figure 6:** Flowchart of DE-BP model.

**Figure 7:** Convergence curve of DE optimization algorithm.

**Figure 8:** Prediction results of 100M run.

**Figure 9:** General test results.

**Table 1:** Prediction accuracy of different models.

Model	Prediction accuracy (%)	RMSE	MAPE (%)
Multiple linear regression	86.78	0.3217	6.646
GA-BP	89.12	0.2413	5.241
PSO-BP	89.86	0.1674	3.471
DE-BP	92.31	0.0758	2.529

## Data Availability

The dataset can be accessed upon request.
